# Effects of Aerobic Exercise on the Serum Leptin Level and Heart Rate Variability in the Obese Girl Children

**DOI:** 10.1155/2022/2298994

**Published:** 2022-06-10

**Authors:** Cuihan Li, Shaojun Lyu, Jianwei Zhang

**Affiliations:** College of P.E. and Sports, Beijing Normal University, Beijing 100875, China

## Abstract

**Objective:**

The present study examined the effects of a 16-week aerobic exercise (AE) on the serum leptin level and heart rate variability (time domain and frequency domain) in the obese girl children and correlation coefficients of changes between the serum leptin level and heart rate variability after a 16-week AE intervention.

**Methods:**

36 participants were randomly assigned to either aerobic exercise (AE, *n* = 18) or obese group (*n* = 18). The obese girl children in the AE group conducted a 16-week (4 times per week and 60 min per time) exercise protocols, and the obese group did not perform regular physical training during 16 weeks of study. Then, the serum leptin level and HRV (time domain and frequency domain) were measured in all subjects before and after AE intervention.

**Results:**

(1) After 16-week AE intervention, compared with pre-exercise, LF/HF decreased (*P* < 0.05), HF, SDNN, and RMSSD significantly increased (*P* < 0.05 and *P* < 0.01), and there was no significant difference in LF (*P* > 0.05) in the AE group. Nevertheless, there was no significant change before and after the test in the serum leptin level and HRV of the obese group (*P* > 0.05, respectively). (2) After 16-week AE intervention, compared with the obese group, SDNN and HF significantly increased (*P* < 0.05, respectively), LF/HF significantly decreased (*P* < 0.05) in the AE group, but there was no significant difference in RMSSD and LF between the obese group and AE group. (3) The reduction variables of the serum leptin level before and after the AE intervention are positively correlated with the reduction in the LF/HF (*r* = 0.478, *P* < 0.05) and negatively correlated with the increasing in the RMSSD (*r* = −0.482, *P* < 0.05). But there is no significant association between the reduction in the serum leptin level and the change of LF, HF, and SDNN (*P* > 0.05, respectively).

**Conclusion:**

16-week AE significantly reduced the serum leptin level and improved cardiac autonomic function in the obese girl children. Moreover, the reduction in the serum leptin level was associated with the increase in parasympathetic activation and improved sympathetic-vagus balance after AE intervention. More research is needed to see whether the effect of exercise on leptin levels in obese girl children can reduce the risk of cardiovascular disease in adulthood.

## 1. Introduction

With economic development and improvement of living standards, the number of children with obesity is rapidly increasing around the world, which seriously affects the children's growth, development, and physical and mental health. Studies suggest that obesity increases the risk of cardiovascular disease; moreover, dysregulation of autonomic nerve function (ANS) is one of the potential mechanisms and causes the changes in cardiometabolism of obese patients [1]. In addition, ANS is an important system of regulating energy balance and plays an important role in the pathophysiology of obesity [2]. Therefore, ANS has important clinical significance in the study of obesity patients. Heart rate variability (HRV) has been recognized as a quantitative measure for noninvasive assessment of cardiac autonomic regulation (cardiac, parasympathetic, and sympathetic). Knutson et al. [3] found that obese children showed the sympathovagal dysregulation and lower heart rate variability than normal-weight children. Another study found that overweight and/or obese children showed the sympathetic hyperactivity and decreased the parasympathetic function when compared with normal-weight children, especially at night [4]. Therefore, it is crucial to balance the activity of the sympathovagal nervous system in obese patients. Most studies have shown that regular exercise can enhance vagus nerve activity in obese patients which contribute to reduce the risk of cardiovascular disease and sudden cardiac death [5], but the mechanism is unclear.

Leptin is a 16 kDa peptide hormone and mainly derives from adipose tissue which suppresses appetite, increases energy expenditure, and reduces body weight by acting its receptors in the hypothalamus [6]. Studies have shown that overweight and obese patients have higher leptin concentrations, and most obese individuals exist “leptin resistance” [7]. In addition, elevated leptin levels have been shown to be directly associated with systemic inflammation, immune-mediated disease, cerebrovascular and cardiovascular disease, and it can lead to the autonomic dysregulation. Charles et al. [8] found that leptin levels were significantly negatively correlated with HRV, especially among officers with higher body weight (BMI ≥25 kg/m^2^) through a study of 388 public security personnel, which suggested that elevated leptin levels may be associated with cardiovascular disease. And, animal studies have shown that the increasing leptin level on sympathetic nerve activity was dose-dependent, and it could lead to autonomic dysfunction and was associated with cardiovascular morbidity and mortality [9]. Therefore, it may be considered that leptin may play an important role in sympathovagal imbalance of obese children. Meta-analysis showed that regular exercise, especially aerobic exercise, can significantly reduce serum leptin levels in obese children [10]. And, scholars have found that aerobic exercise intervention has been shown to improve cardiac automatic rhythm function in adults and children [11]. However, there are few studies on whether the improvement of cardiac autonomic regulation in obese children by aerobic exercise is related to the decrease of serum leptin. Therefore, the present study examined the effects of a 16-week aerobic exercise (AE) on the serum leptin level and heart rate variability (time domain and frequency domain) in the obese girl children and determined whether these effects were related to changes in serum leptin levels in order to provide a theoretical basis for aerobic exercise to improve cardiovascular health in obese children.

## 2. Research Objects and Methods

### 2.1. Subjects

According to the standard height and weight value of Chinese students aged 7–22, those whose actual weight is more than 20% of the standard weight are regarded as obese, mildly obese (20–29% overweight), moderately obese (30–49% overweight), and more than 50% were severely obese [12]. According to the above criteria, 36 obese female children from Affiliated Primary School of Beijing Normal University were recruited. The subjects were all simple obesity and were randomly divided into obesity group (*n* = 18) and aerobic exercise group (*n* = 18). As shown in Table 1, there was no significant difference in age, height, weight, and BMI between the two groups by independent samples *T*-test (all *P* > 0.05).

#### 2.1.1. Inclusion Criteria

The subjects who had been diagnosed without hypertension, diabetes, dyslipidemia, and cardiovascular disease or who were not consuming weight-reducing medicine or no regular exercise program or physical activity in the past 3 months were included. All participants and their parents or guardians were informed of the purpose of the experiment and voluntarily participated in the exercise training and signed informed consent before training.

### 2.2. Research Methods

#### 2.2.1. Aerobic Exercise Program [10]

From March to July in 2020, obese female children in the aerobic exercise group were given 16 weeks of aerobic exercise (badminton, aerobics, jogging, power cycling, and sports games), 4 times a week, each exercise for 60 minutes (warm up for 5 minutes, formal training for 50 minutes, and relaxation training for 5 minutes), and exercise intensity of 220-age × 65%–70%; the whole training process is guided by professional physical education teachers, and the exercise intensity is supervised by polar table.

#### 2.2.2. HRV Indicator Evaluation

Before and after the exercise intervention, the subjects wore the heart rate of Polar Team 2 (made in Finland) and measured the HRV of subjects. After the height, weight, date of birth, and other information were put into the computer of the subjects and rest 5 min with eyes closed in a quiet environment. Subsequently, the heart rate for 10 min(10 subjects for each test) was recorded, and then the Kubios HRV software is used to calculate the HRV time domain and frequency domain indicators.

Time domain indexes include SDNN (standard deviation of all R-R intervals, ms) and RMSSD (square root of the sum of the mean of the difference between adjacent RR intervals, ms). Frequency domain indicators include low frequency power (LF, 0.04–0.15 Hz; sympathetic activity index) and high frequency power (HF, 0.15–0.40 Hz; vagus nerve activity level index) and LF/HF ratio (sympathetic-vagus nerve balance index).

#### 2.2.3. Measurement of the Blood Leptin Level

Before and after the exercise intervention, blood samples from all subjects were collected at our laboratory at 08:00 following a 12-hour overnight fast. After a 10-minute rest in a comfortable chair, fasting blood was collected from the median cubital vein into a plain tube. Each blood sample was centrifuged at 3,000 g for 10 minutes at 4^o^C, and serum leptin levels were determined by radioimmunoassay (according to the instructions).

### 2.3. Data Analysis

All experimental data were expressed as mean ± standard deviation, and the data were analyzed using SPSS 19.0. All experimental data belonged to the normal distribution by K–S test. Paired *t*-test was used to compare the differences in the levels of leptin and HRV parameters before and after the experiment, and independent samples *t*-test was used to compare the differences in the above data between obese group and aerobic exercise group. The correlation of the changes in serum leptin levels and HRV parameters after aerobic exercise intervention was analyzed by Pearson correlation, and a *P* value of 0.05 indicated that the difference was considered statistically significant.

## 3. Research Results

### 3.1. The Effect of Aerobic Exercise on Serum Leptin Level in Obese Female Children

As shown in Table 2, after 16 weeks of aerobic exercise intervention, compared with pre-exercise, the serum leptin level of the obese exercise group significantly decreased (*P* < 0.01) by 13.06%. Independent sample *T*-test showed that there was no significant difference in serum leptin level between the obese group and the obese exercise group before aerobic exercise intervention (*t* = -0.155, *P* = 0.878). After 16 weeks of aerobic exercise, compared with the obese group, the serum leptin level in the obese exercise group significantly decreased by 15.21% (*t* = 2.645, *P* = 0.012).

### 3.2. Effects of Aerobic Exercise on HRV in Obese Female Children

As shown in Table 3, after 12 weeks of aerobic exercise intervention, SDNN and RMSSD in the obese exercise group significantly increased compared with those pre-exercise (all *P* < 0.01); The frequency domain index LF/HF significantly decreased, and HF significantly increased (*P* < 0.05). There was no significant change in LF before and after exercise intervention (*P* > 0.05). There was no significant difference in the above indicators in the obese group before and after the experiment (all *P* > 0.05).

Independent sample *T* test showed that there was no significant difference in HRV parameters between the two groups before aerobic exercise intervention (all *P* > 0.05). After 16-week aerobic exercise, compared with the obese group, SDNN of HRV time domain index significantly increased (*t* = −2.641, *P* = 0.012) in the obese exercise group. There was no significant difference in RMSSD and frequency domain LF (*t* = −0.783, *P* = 0.439; *t* = −0.103, *P* = 0.918) between the two groups. While LF/HF in the obese exercise group was significantly lower than that of the obese group (*t* = 2.334, *P* = 0.026), and HF was significantly higher than that of the obese group (*t* = −2.111, *P* = 0.045).

### 3.3. Correlation Analysis between Changes in Serum Leptin Levels and HRV Parameters after Aerobic Exercise Intervention

As shown in Table 4, Pearson correlation analysis showed that, after 16 weeks of aerobic exercise intervention, the change of serum leptin was significantly negatively correlated with the change of HRV time domain index RMSSD (*r* = −0.482 *P* < 0.05) and significantly positively correlated with the change of HRV frequency domain index LF/HF (*r* = 0.512, *r* = 0.478, *P* < 0.05). There was no significant correlation with the changes of LF, HF, and SDNN (all *P* > 0.05).

## 4. Discussion

### 4.1. The Effect of Aerobic Exercise on HRV in Obese Female Children

Studies suggest that cardiovascular risk factors such as hyperglycemia, hypertension, and abnormal plasma lipoprotein levels in obese children which increase the likelihood of developing atherosclerotic cardiovascular disease in adulthood, and changes of ANS play an important role in the pathogenesis of these diseases [13]. HRV has emerged as a reliable noninvasive method to assess ANS activity, especially SDNN can reflect the overall activity of ANS. Low frequency (LF) is mainly mediated by sympathetic activity, and RMSSD and HF are associated with vagal activity [14]. Prior study found that compared with normal weight children (BMI: 17.7 ± 2.8 kg/m^2^) and obese children (11.6 ± 3.8 years old; BMI: 29.8 ± 4.6 kg/m^2^), the heart rate variability indicators SDNN, RMSSD, and pNN50 significantly decreased in the obese group which suggested that obesity may lead to sympathovagal imbalance or disorder and increase the risk of cardiovascular disease in obese children [15]. Paschoal et al. [16] found that compared with normal-weight children (10.2 ± 0.7 years), HRV frequency domain indicators LFn and LF/HF ratio significantly decreased and HFn significantly increased in the standing position of the obese children, indicating that cardiac sympathetic nerve activity was enhanced and parasympathetic nerve activity was weakened. Therefore, improvement of ANS activity is critical in obese children. The prior study found that the level of physical exercise can affect the cardiac autonomic function, and the study showed that regular exercise increased the HF of obese children, while the decreasing of RMSSD stopped after exercise, indicating that regular physical exercise had a good effect on the parasympathetic (vagus) activity of obese children [17]. However, the conclusion that physical exercise improving ANS in obese children is inconsistent. Gutin et al. [18] conducted a 12-month moderate-intensity exercise intervention (5 days/week, 20 min each time, heart rate 130–140 bpm) in obese children (6–11 years old) and found that exercise significantly increased HF and decreased LF in obese children, which suggested that moderate-intensity physical activity improves sympathetic and vagal activity in obese children. And, LI [19] found that Taijiquan exercise can improve the integration and regulation function of cardiac autonomic nerve, especially vagus nerve activity. In addition, Biljon et al. [20] found that moderate-intensity aerobic exercise (exercise intensity: 65–70% HRmax) might increase vagal activity (increasing in HF) in normal-weight children (11.07 ± 0.81 years) and cause sympathovagal balance (ratio of LF/HF decreasing) which seemed to induce superior alterations in cardiac ANS activity in normal-weight children. Mandigout et al. [21] conducted a 13-week endurance training program (exercise intensity >80% HRmax) in 19 obese children (10–11 years old) and found that LF and HF of obese children after endurance training were significantly higher than those before training, but the LF/HF ratio did not significantly change. The results showed that endurance training had a positive effect on HRV in healthy children, but did not induce sympathetic and parasympathetic modifications. The results of current study are consistent with previous studies that the moderate-intensity exercise program improves the HRV in obese children. The results of current study shows that time domain indicators SDNN and RMSSD significantly increased, the frequency domain HF increased, the ratio of LF/HF decreased, but LF did not significantly change in the obese exercise group when compared with the obese children group which indicated that physical exercise can increase heart rate variability and stimulate vagal tone, but has no effect on sympathetic nerve activity. Different results are obtained for different studies, which may be related to different exercise time, intensity, and research objects.

### 4.2. The Effect of Aerobic Exercise on the Serum Leptin Level in Obese Female Children

Leptin reduces food intake and increases the activity of the sympathetic nervous system by acting relevant receptors in the hypothalamus. It can reduce fatty acid (FFA) and lipid synthesis and also directly act on adipocytes in the body to inhibit fat synthesis. It plays an important role in body weight regulation and leptin resistance in overweight and obese individuals, and it plays an important factor in weight control [22]. And, studies suggest that there is a positive correlation between circulating leptin levels and greater future BMI or body adiposity, which can predict the risk of future obesity in children [23], so lowering leptin levels is crucial for obese children. Most scholars believe that the reduction of body fat is the main reason that exercise affects leptin levels, and Willis et al. [24] found that compared with resistance training and resistance training combined with aerobic exercise, aerobic exercise is considered to be the best way to reduce body fat, but the effect on serum leptin levels is more controversial. Meta-analysis showed that physical exercise can increase adiponectin, reduce the plasma levels of leptin and IL-6, and significantly improve the inflammatory status of obese children without changing dietary habits or other lifestyles [10]. And, Zhang et al. [25] thought that long-term Taijiquan practice reduced the concentration of blood-insulin and leptin, promote the fat catabolism, and was helpful for health, fitness, and losing weight. However, Zguira et al. [26] conducted 8 weeks (90 min, 3 days/week) training on obese patients with metabolic syndrome (14 ± 2 years) and found that serum leptin level did not significantly change before and after exercise. The results of this study are the same as those of the former study. After 16 weeks of aerobic exercise intervention, compared with the obese children, the serum leptin level of the obese exercise group significantly decreased. Zhiping et al. [27] believed that the decrease in leptin concentration after aerobic exercise intervention may be related to the reduction of body fat and the negative energy balance caused by exercise training; and García-Hermoso et al. [28] believed that the longer the exercise time (≧60 min), the higher the energy expenditure (≧800 kcal) and the lower the leptin concentration which indicated that the duration of exercise training and the time of every exercise training were significantly negatively correlated with the leptin level. Therefore, it can be considered that the decreasing of serum leptin level in obese children after 16-week aerobic exercise intervention in this study may be related to the reduction of body fat in obese children, and the different changes in the leptin level after exercise intervention may be related to exercise training time and exercise training intensity.

### 4.3. Correlation Analysis of the Serum Leptin Level and Heart Rate Variability

Studies suggested that leptin is independently correlated with different markers of autonomic nervous activity [29]. In addition, Paolisso et al. [30] found that leptin is positively correlated with heart rate variability index LF and LF/HF ratio in 120 normal males (42.5 ± 1.9 years old), which reflected that leptin level is closely correlated with the increasing sympathetic nervous activity. The same results were obtained in adult women (20.9 ± 0.33 years old) by Flanagan et al. [31]. There was a positive correlation between the leptin level and LF or LF/HF in adult women, and the leptin level had a greater impact on the sympathetic nervous system of women with high body fat. However, there was no significant correlation between LF or LF/HF in males (20.9 ± 0.22 years). Wielle [32] found that the serum leptin level was significantly positively correlated with LF or LF/HF in male and female children and negatively correlated with parasympathetic activity (HF and pNN50) in male children, but without significantly associated with parasympathetic activity in female children through follow-up (6.7–12.2 y) study of children (4.4 to 11.0 years old). In the current study, correlation analysis showed that the decreased level of serum leptin was significantly positively correlated with the decrease in HRV frequency domain index LF/HF, but not with the change of LF and HF before and after aerobic exercise intervention in obese female children. This study also found a significant negative correlation between decreased serum leptin level and increased RMSSD, suggesting a significant negative correlation between serum leptin level and parasympathetic neural activity in female children, which is different from the above results. Umetani et al. [33] believe that HRV is related to gender and age. Therefore, it can be considered that the difference between our study, and the above research results may be related to the selection of research objects.

## Figures and Tables

**Table 1:** Basic information of the objects $\left(\bar{x}\pm s\right)$.

Group	Age	Height (m)	Weight (kg)	BMI (kg/m^2^)
Obese group	11.58 ± 0.27	1.53 ± 3.02	58.12 ± 2.64	24.12 ± 3.08
Aerobic exercise group	12.04 ± 0.96	1.54 ± 4.12	58.86 ± 2.82	24.59 ± 3.36
*P*	0.098	0.078	0.063	0.096

**Table 2:** Results of the serum leptin level in each group of obese female children $\left(\bar{x}\pm s\right)$.

Group	*n*	Before serum leptin level, *μ*g/L	After serum leptin level, *μ*g/L	*t* value	*P* value
Obese group	18	21.83 ± 3.73	22.61 ± 3.18	−1.740	0.100
Aerobic exercise group	18	22.05 ± 4.80	19.17 ± 4.51^ΔΔ#^	10.363	0.000

*Note.* ^Δ^ *P* < 0.05 and ^ΔΔ^*P* < 0.01, comparison before and after the experiment; ^#^*P* < 0.05, comparison between obese group and obese exercise group.

**Table 3:** Results of the HRV in each group of obese female children $\left(\bar{x}\pm s\right)$.

HRV	Group	Before	After	*T* value	*P* value
SDNN (ms)	Obese group	126.67 ± 13.05	128.89 ± 10.72	−0.885	0.388
	Obese exercise group	128.88 ± 10.72	139.67 ± 13.59^ΔΔ#^	−10.361	0.000

RMSSD (ms)	Obese group	46.06 ± 8.33	46.89 ± 8.33	−0.995	0.334
	Obese exercise group	45.17 ± 8.83	49.28 ± 8.86^ΔΔ^	−10.719	0.000

LF (ms^2^)	Obese group	1026.67 ± 424.51	1008.44 ± 396.05	0.663	0.516
	Obese exercise group	1078.39 ± 474.39	1023.94 ± 497.93	1.831	0.085

HF (ms^2^)	Obese group	677.71 ± 304.81	645.03 ± 303.79	0.386	0.705
	Obese exercise group	697.09 ± 306.98	986.03 ± 614.45^Δ#^	−2.728	0.014

LF/HF	Obese group	1.73 ± 0.86	1.74 ± 0.75	−0.065	0.949
	Obese exercise group	1.79 ± 1.09	1.20 ± 0.63^Δ#^	2.706	0.015

*Note.* ^Δ^ *P* < 0.05 and ^ΔΔ^*P* < 0.01, comparison before and after the experiment; ^#^*P* < 0.05, comparison between obese group and obese exercise group.

**Table 4:** Correlation coefﬁcients (*r*) of changes between serum leptin level and heart rate variability after a 16-week aerobic exercise intervention $\left(\bar{x}\pm s\right)$.

		ΔHF (ms^2^)	ΔLF (ms^2^)	ΔLF/HF	ΔSDNN (ms)	ΔRMSSD (ms)
Δ serum leptin level (*μ*g/L)	r	−0.070	0.159	0.478^*∗*^	0.258	−0.482*∗*
	*P*	0.782	0.530	0.046	0.301	0.043

## Data Availability

The experimental data used to support the findings of this study are available from the corresponding author upon request.

## Additional Points

16-week aerobic exercise significantly reduced serum leptin level and improved cardiac autonomic function in obese female children, and the decreasing of serum leptin concentration after aerobic exercise intervention was associated with the increasing of sympathetic vagus nerve balance to parasympathetic nerve activity. But more research is needed to confirm whether the effect of exercise on leptin levels in obese female children can reduce the risk of cardiovascular disease in adulthood.
